RETRACTED

# HOXC10 Promotes the Metastasis of Human Lung Adenocarcinoma and Indicates Poor Survival Outcome

**DOI:** 10.3389/fphys.2017.00557

**Published:** 2017-08-02

**Authors:** Xiao-Lei Tang, Bang-Xian Ding, Ying Hua, Hao Chen, Tao Wu, Zhang-Quan Chen, Chun-Hui Yuan

**Affiliations:** ^1^Department of Laboratory and Nuclear Medicine, People's Hospital Anhui, China; ^2^Department of Laboratory Medicine, Wuhan Children's Hospital, Huazhong University of Science and Technology Wuhan, China; ^3^Chemical and Biological Engineer, Vocational and Technical College of Fuyang Anhui, China; ^4^Department of Pathology, Zhongnan Hospital of Wuhan University Wuhan, China; ^5^Key Laboratory for Medical Molecular Diagnostic of Guangdong Province, Guangdong Medical University Dongguan, China

**Keywords:** HOXC10, lung adenocarcinoma, metastasis, invasion, survival

## Abstract

**Background:** As master regulator of embryonic morphogenesis, homeodomain-containing gene 10 (HOXC10) has been found to promote progression of human cancers and indicates poor survival outcome. However, the role of HOXC10 in lung adenocarcinoma still unclear.

**Methods:** HOXC10 expression was evaluated in 63 primary lung adenocarcinoma tissues from our local hospital, and further systematically confirmed in lung cancer tissues from six GEO datasets (GSE19188, GSE31210, GSE10072, GSE7670, GSE32863, GSE30219), and Kaplan-Meier plotter database. The role of HOXC10 in lung cancer metastasis was further validated by cellular and molecular studies.

**Results:** The expression of HOXC10 was significantly increased in human lung adenocarcinoma samples from Wuhu No.2 People's Hospital, about 4.219 times compared with normal tissues, and significantly correlated with TNM stage, lymph node, and distal metastasis. Upregulation of HOXC10 indicated a poor overall/relapse free survival of lung cancer patients from Wuhu No.2 People's Hospital, GEO datasets, and Kaplan-Meier plotter database, especially in patients with lung adenocarcinoma. Knockdown or ectopic expression assays confirmed that HOXC10 enhanced the phosphorylation of PI3K, regulated the expression of epithelial-to-mesenchymal transition (EMT) markers: MMP2/9, VCAM-1, vimentin and E-cadherin. Cellular study further confirmed that HOXC10 was required for migration, invasion and adhesion of lung cancer cells.

**Conclusion:** These findings suggest that HOXC10 plays a pivotal role in the metastasis of human lung cancer and highlight its usefulness as a potential prognostic marker or therapeutic target in human lung adenocarcinoma.

## Introduction

Lung cancer is the foremost cause of cancer-related death worldwide. The two types of lung cancer are non-small-cell lung cancers (NSCLCs; 80% of all lung cancers), and small-cell lung cancers (20%, exhibiting neuroendocrine features) (Imielinski et al., 2012). NSCLC has a very poor prognosis and the average five-year survival rate is approximately 15% (Ma et al., 2015), principally because it is most commonly diagnosed at an advanced stage, and usually accompanied with aggressive local invasion, regional lymph node or distant metastasis (Forde and Ettinger, 2013; Yang et al., 2014). However, surgery or therapies that treat primary lung tumors rarely prevent metastasis (Siegel et al., 2013). Thus, to further understand the mechanisms of lung cancer metastasis is crucial for the development of new therapies to improve survival for lung cancer patients.

RETRACTED

There are 39 homeobox (HOX) genes organized into four different genomic clusters (*HOX A-D*) located on four chromosomes (7, 17, 12, and 2) of humans (Alexander et al., 2009). HOX genes are highly conserved at the genomic level and have been well-described as important players in regulating numerous processes including apoptosis, receptor signaling, differentiation, motility, angiogenesis, and metastasis (Grier et al., 2005; Shah and Sukumar, 2010). Aberrations in HOX gene expression have been reported in numerous malignancies, including ovarian cancer (Morgan et al., 2010), esophageal squamous cell carcinoma (Chen et al., 2005), breast cancer (Pathiraja et al., 2014), lung cancer (Calvo et al., 2000; Plowright et al., 2009), gastric cancer (Yuan et al., 2016) and hematological malignancies (Argiropoulos and Humphries, 2007), and significantly enhanced invasiveness, proliferation and colony formation of tumor cells (Ma et al., 2003; Wu et al., 2006; Miao et al., 2007). In lung cancers, about 20–25 HOX genes are expressed at least two-fold higher than normal tissues (Tiberio et al., 1994; Calvo et al., 2000; Plowright et al., 2009), especially, homeobox gene HOXD3 upregulation induced coordinate expression of metastasis-related genes in human lung cancer cells (Hamada et al., 2001), these results indicated that HOX genes could provide new targets for future tumor therapies.

HOXC10, as a member of HOX genes family, significantly enhances the proliferation, invasion and metastasis of cancer cells, and may be useful as marker for cancer diagnosis or progression evaluation (Gabellini et al., 2003; Zhai et al., 2007; Feng et al., 2015). In cervical squamous cell carcinomas, elevated HOXC10 expression was associated with increased invasiveness as identified by using high-density oligonucleotide microarrays (Zhai et al., 2007). In the Cancer Genome Atlas (TCGA) datasets, HOXC10 expression was significantly increased in human thyroid cancer tissues when compared with normal human thyroid tissues (Feng et al., 2015). Furthermore, HOXC10 promoted migration and invasion of thyroid cancer cells, and has the potential to be a novel biomarker for human thyroid cancer prognosis (Feng et al., 2015). However, the role of HOXC10 in breast cancer remains controversial. Two separate studies conducted by Sadik (Sadik et al., 2016) and Khairul (Ansari et al., 2012) found that HOXC10 is transcriptionally regulated by estrogen and overexpressed in primary carcinomas of the breast, and even more significantly in distant metastasis arising after failed chemotherapy, but in another study conducted by Pathiraja et al. (2014) reported that HOXC10 expression was repressed by estrogen and decreased in breast cancer tissues.

RETRACTED

Despite these clues suggest that HOXC10 regulates metastasis-related activities in other tumor types, the role of HOXC10 in lung cancer metastasis remains unclear. In this study, we determined that HOXC10 expression is significantly increased in human lung cancer tissues compared with normal human lung tissues, and its overexpression expression is significantly correlated with TNM stage, lymph node and distal metastasis, as well as poor overall survival. Knockdown or ectopic expression assays further confirmed that HOXC10 was required for migration, invasion and adhesion of lung cancer cells. In addition, HOXC10 is significantly upregulated and indicates poor survival in lung cancer by mining clinical and expression profile from GEO Datasets and Kaplan-Meier plotter database. Therefore, our work demonstrates that HOXC10 enhances the metastasis of human lung cancer cells, and which might be a potential target for treatment of lung cancer and a marker for prognosis of lung cancer patients.

## Materials and methods

### Patients and tissue samples

The study was approved by the ethics committee of Wuhu No.2 People's Hospital and informed consent was obtained from all participated patients. Sixty three lung adenocarcinoma tissues and 30 non-cancerous tissues were obtained from Department of pathology, Wuhu No.2 People's Hospital. Clinicopathologic characteristics of all patients (Table 1) were also collected, and none of these patients had received local, systemic treatments or surgical treatment before biopsy. Tissue samples were immediately snap-frozen in liquid nitrogen and stored at −80°C until total RNA or protein was extracted. Tumor samples were composed of at least 80% viable appearing tumor cells on histological assessment.

**Table 1:** Clinicopathologic characteristics of lung cancer patients.

**Characteristics**	**Cases (%)^#^**	**HOXC10 mRNA expression (Mean ± SD)**	***p*-value**
Total	63	4.219 ± 2.134	
Gender			0.6330
Male	41 (65.1)	4.124 ± 2.168	
Female	22 (34.9)	4.396 ± 2.108	
Age (years)			0.3293
≥60	43 (68.3)	4.058 ± 1.969	
< 60	20 (31.7)	4.654 ± 2.544	
Tumor size (longest dimension) ≤ 5 cm	49 (77.7)	4.188 ± 2.094	0.8312
>5 cm	14 (22.3)	4.327 ± 2.347	
Smoking status			0.0031^*^
Current or former smoker	45 (71.4)	4.710 ± 2.148	
Non-smoker	18 (28.6)	2.990 ± 1.559	
TNM stage			< 0.0001^*^
I-II	25 (39.7)	2.955 ± 1.196	
III-IV	38 (60.3)	5.050 ± 2.217	
Lymph node Metastasis			< 0.0001^*^
N0	40 (63.5)	2.975 ± 1.458	
N1-3	23 (36.5)	4.934 ± 2.146	
Distal metastasis			< 0.0001^*^
M0	46 (73.0)	3.605 ± 1.407	
M1	17 (27.0)	5.879 ± 2.840	

*TNM, tumor-node-metastasis; SD, Standard deviation*.

* *p < 0.05 was considered statistically significant*.

RETRACTED

# *Three patients were excluded in survival analysis as information missed during follow-up*.

### Immunohistochemistry

Tissue samples were fixed in 4% formalin, and embedded in paraffin. Antigen retrieval was enhanced by microwaving the slides in citrate buffer (pH 6.0) for 10 min. Sections were incubated with rabbit polyclonal anti-HOXC10 (1:500 dilution, Abcam) overnight at 4°C. Antigen-antibody complexes were detected with the avidin-biotin peroxidase method using 3,3′—diaminobenzidine as a chromogenic substrate (DAB kit, ZSGB-Biotechnology Co., Ltd, Beijing, China). Sections were lightly counterstained with hematoxylin and examined by light microscopy.

### Cell culture

The human lung adenocarcinoma cell lines (H1975, PC-9, A549), Large cell lung cancer cell (H460), small cell lung cancer cell (H446), and the normal lung cell (MRC5) were obtained from Academia Sinica Cell Bank (Shanghai, China). Except for MRC5 was cultured in MEM, all the other cell lines were maintained in DMEM (Life Technologies, CA, USA), supplemented with 10% fetal bovine serum (FBS, Life Technologies), 100 U/mL penicillin, and 100 μg/mL streptomycin (Beyotime, Shanghai, China), in a humidified atmosphere at 37°C with 5% CO_2_. The cells in the exponential phase of growth were used in the experiments.

### Cell transfection

Short hairpin RNA (shRNA) for HOXC10 (20 nM) and scramble shRNA control were obtained from Genesil Biotechnology (Wuhan, China). shRNA targeting position 830–852 (CGGAUAACGAAGCGAAAGA; named HOXC10 shRNA) of human HOXC10 mRNA was cloned into a lentiviral vector (PLKO.1-C1). HOXC10 mRNA (GenBank accession no. NM_017409.3) was amplified from normal human lung tissue and inserted into the pcDNA3.1 vector (Invitrogen, Carlsbad, CA, USA). The transfection of H1975 and H460 cells were performed with Lipofectamine 2000 (Invitrogen, Shanghai, China) following the manufacturer's protocol. Scramble shRNA control and empty vector were used as negative control (NC), respectively. 48 h after transfection, the selective silencing and overexpression of HOXC10 were identified by quantitative Real-Time PCR (qRT-PCR) and western blotting analysis.

RETRACTED

### Quantitative real-time PCR (qRT-PCR)

Total RNAs from tissue samples and cells were isolated with TRIZOL reagent (Life Technologies) according to the manufacturer's instruction. Total RNA (1 μg) was reversely transcribed into cDNA using RevertAid First Strand cDNA Synthesis Kit (ThermoFisher Scientific, Waltham, MA) with the oligo-dT primer. qRT-PCR was performed with Maxima SYBR Green/ROX qPCR Master Mix (ThermoFisher Scientific) according to the manufacturer's instructions to detect mRNA levels of indicated genes. The primers used were as follows: HOXC10 (Forward: 5′—GCTTGA AGTCTCGTATTTG-3′, Reverse: 5′-CTGTCTTTGCTTTGCTATG-3′), matrix metallopeptidase 2 (MMP2) (Forward: 5′-TTGACGGTAAGGACGGACTC-3′, Reverse: 5′-GGCGTTCCCATACTTCACAC-3′), MMP9 (Forward: 5′-AAGGGCGT CGTGGTTCCAACTC-3′, Reverse: 5′-AGCATTGCCGTCCTGGGTGTAG-3′), E-cadherin (Forward: 5′-GAGAACGCATTGCCACATACAC-3 ′, Reverse: 5′-AAGAG CACCTTCCATGACAGAC-3′), vascular cell adhesion molecule 1 (VCAM1) (Forward: 5′-TGGGAACGAACACTCTTAC-3′, Reverse: 5′-CAGCAACTGAACA CTTGAC-3′), vimentin (Forward: 5′-GACAATGCGTCTCTGGCACGTCTT-3′, Reverse: 5′-AAGAACCTGCAGGAGGCAGAAGAA-3′), GAPDH (Forward: 5′-CA CCCACTCCTCCACCTTTG-3′, Reverse: 5′-CCACCACCCTGTTGCTGTAG-3′). The ABI 7300 (Applied Biosystems, CA, USA) was used to perform the amplification reaction. Each experiment was performed in triplicate. And the date was analyzed by the 2^−ΔΔCt^ method (Chen et al., 2016).

### Western blotting analysis

Thirty microgram of total protein were loaded on 10% SDS-PAGE using a Bio-Rad miniature slab gel apparatus and electrophoretically transferred onto PVDF membranes. Membranes were blocked with 5% skimmed milk and incubated overnight at 4°C with primary antibodies. Primary antibodies against HOXC10, MMP-2, MMP-9, and VCAM-1 were purchased from Abcam (Cambridge, MA, USA). Antibody for JNK, phospho-JNK, ERK1/2, phospho-ERK1/2, PI3K, phospho-PI3K, E-cadherin, and GAPDH were from Cell Signaling Technology, Inc. (Beverley, MA, USA). Target proteins were visualized by enhanced chemiluminescence (Millipore, Beijing, China) according to the manufacturer's instructions.

### Migration assay

H1975 and H460 cells were firstly transfected with HOXC10 shRNA and pcDNA3.1-HOXC10, respectively. 48 h later, cells were trypsinized and resuspended in DMEM with 1% FBS. Then 5 × 10^4^ cells were transferred on the top chambers (8-μm pore size, Corning Costar) of 24-well-plate. Ten percent FBS-medium were added in the lower chamber and incubated for 48 h. Cells were fixed with 4% methanol for 15 min and then stained with 0.5% crystal violet for 30 min. The numbers of invaded cells at the lower membrane side were counted under microscope, and three random fields were scanned. Experiments were performed in three independent times.

RETRACTED

### Invasion assay

H1975 and H460 cells were pretreated similar with migration assay. Transwell chambers were precoated with 80 μL matrigel (2.5 mg/ml; BD, CA, USA) and incubated at 37°C for 30 min according to the manufacturer's instructions. Next, the transwell chambers coated with Matrigel were used for invasion assay. A total of 5 × 10^4^ cells in 1% FBS-DMEM were placed in the upper chamber and 10% FBS-DMEM were added in the lower chamber. After 48 h incubation, the cells that had invaded another side of the membrane were fixed with methanol for 15 min and then stained with 0.5% crystal violet for 30 min. The numbers of invasive cells were counted under microscope.

### Adhesion assay

H1975 and H460 cells were pretreated similar with migration or invasion assay. 12-well plates were precoated with 10 μg/ml of fibronectin and incubated at 37°C for 2 h (Mahauad-Fernandez et al., 2014). Non-specific sites were blocked with 40 μl of 2 mg/ml bovine serum albumin (BSA) in PBS. Wells were washed once with PBS. A total of 2 × 10^4^ cells were added to the plate and allowed to attach for 60 min. Then plates were washed with PBS to remove non-adhered cells. Attached cells were fixed with 4% paraformaldehyde for 15min and then stained with 0.5% crystal violet for 30 min. The numbers of attached cells were counted under microscope. Experiments were performed in three independent times.

### Statistical analysis

All data are presented as mean ± SD and analyzed by using the Graphpad Prism V.5.00 software (GraphPad Software, CA, USA). Comparison between two groups for statistical significance were performed with unpaired Student's *t*-test. For more groups, one-way ANOVA followed by Neuman-Keuls *post-hoc* test was used. Survival analysis was carried out by the Kaplan-Meier method, and subjected to the log rank test. *P* < 0.05 was considered statistically significant.

## Results

### HOXC10 is overexpressed in human lung cancer tissues

To determine whether HOXC10 was involved in lung cancer progression, we firstly examined mRNA level of HOXC10 in cancer and adjacent normal tissues from patients with lung adenocarcinoma in Wuhu No.2 People's Hospital. mRNA level of HOXC10 in lung adenocarcinoma tissues was significantly higher than normal lung tissues, about 4.219 times over normal tissues as identified by qRT-PCR analysis (Figure 1A). Western blotting analysis further showed that the protein expression of HOXC10 was also enhanced in tumor samples (Figures 1B,C). To evaluate the clinical significance of HOXC10, we then assessed the correlation of its expression with clinicopathological characteristics (i.e., smoking status, tumor size, TNM stage and metastasis). As shown in Table 1, HOXC10 mRNA expression was significantly associated with smoking status (*p* = 0.0031), TNM stage (*p* < 0.0001), lymph node metastasis (*p* < 0.0001, Figure 1D) and distal metastasis (*p* < 0.0001, Figure 1E) in lung cancer. In addition, immunohistochemistry analysis further showed that HOXC10 protein levels were significantly elevated in lung adenocarcinoma patients with lymph node or distal metastasis (both in primary site and brain metastasis) than those without metastasis (Figure 1F).

RETRACTED

**Figure 1:** HOXC10 upregulates in human lung cancer tissues. **(A)** Relative mRNA expression of HOXC10 in human lung cancer (*n* = 63) and normal (*n* = 30) tissues was detected by qRT-PCR, GAPDH was used as internal control. **(B)** Protein expression of HOXC10 in tissues from four represent patients was detected by western blotting; and relative HOXC10 expression was normalized to housekeeping gene GAPDH **(C)**. **(D,E)** Data was derived from **(A)**, patients were subdivided into two groups according to lymph node **(D**, N0 and N1-3) or distal metastasis **(E**, M0 and M1), relative mRNA expression of HOXC10 was compared between these two groups, respectively. **(F)** The protein expression of HOXC10 in lung cancer tissues with or without metastasis was evaluated by immunohistochemistry. **(G)** Patients were subdivided into two groups according to the mean value of HOXC10 mRNA expression (cutoff value: 4.219), and survival analysis carried out by the Kaplan-Meier method, and subjected to the log rank test. Data are presented as means ± *SD*, ^***^p < 0.0001.

Next, we divided the patients with lung adenocarcinoma into two groups using a median value of HOXC10 mRNA expression, 4.219 (Figure 1A), and then compared the overall survival time of patients with lung adenocarcinoma. As shown in Figure 1G, the cumulative survival rate was significantly lower in the high HOXC10 expression group (30.8%) compared with the low HOXC10 group (64.7%) (*p* = 0.0033). Thus, these results indicate that HOXC10 may involve in metastasis of lung adenocarcinoma and its expression may represent a new prognostic factor in human lung adenocarcinoma patients.

### Expression of HOXC10 in human lung cancer cell lines

To determine whether HOXC10 was important for metastasis of lung adenocarcinoma cells, we next examined its expression levels in three human lung adenocarcinoma cell lines (H1975, PC-9, A549) and other types of lung cancer cells, H460 and H446, as well as the normal lung cells MRC5. qRT-PCR and western blotting analysis revealed H1975 occupied the highest HOXC10 expression and H460 with the lowest (mRNA and protein levels) (Figures 2A,B; *p* < 0.0001). Therefore, we chose H1975 and H460 cells to explore the role of HOXC10 in lung cancer metastasis, mainly through interfering HOXC10 expression in H1975 cells with HOXC10 shRNA and overexpressing HOXC10 expression with pcDNA3.1-HOXC10 recombinant plasmid in H460 cells.

RETRACTED

**Figure 2:** knockdown or ectopic expression of HOXC10 in human lung cancer cell lines. **(A)** HOXC10 mRNA levels in five lung cancer cell lines and normal lung cells (MRC5). **(B)** HOXC10 protein expressions in these cell lines evaluated by western blotting. Data are presented as means ± *SD, n* = 3, ^***^p < 0.0001 vs. MRC5). **(C)** H1975 cells were untreated or transfected with either HOXC10 shRNA or scramble shRNA control. HOXC10 expression levels were detected by qRT-PCR and western blotting. **(D)** H460 cells were untreated or transfected with either pcDNA3.1-HOXC10 or empty vector. HOXC10 expression levels were detected by qRT-PCR and western blotting. Data are presented as means ± *SD, n* = 3, ^***^p < 0.0001.

The efficacy of the knockdown and overexpression of HOXC10 was examined by Real-time PCR and Western blotting. HOXC10 shRNA significantly decreased mRNA and protein expression of HOXC10 in H1975 cells when compared with scrambled shRNA control (Figure 2C; *p* < 0.0001). In H460 cells, mRNA and protein expression of HOXC10 were significantly enhanced with pcDNA3.1-HOXC10 recombinant plasmid transfection, and no apparent change was observed in the empty vector group (Figure 2D; *p* < 0.0001).

### Effect of HOXC10 on cellular migration, invasion, and adhesion of lung cancer cells

Next, a series of transwell assays were performed to evaluate the influence of HOXC10 on cellular migration and invasion of lung cancer cells. In contrast with untreated or scrambled shRNA control transfected H1975 cells, HOXC10 knockdown significantly decreased the migration and invasion of H1975 cells (Figures 3A,B; *p* < 0.0001). And in H460 cells, HOXC10 ectopic expression markedly enhanced cellular migration and invasion when compared with untreated or empty vector transfected cells (Figures 3C,D; *p* < 0.0001). These results demonstrate that HOXC10 promotes migration and invasion of lung cancer cells from the pros and cons.

**Figure 3:** HOXC10 inhibits cell migration and invasion *in vitro*. H1975 cells and H460 cells were transfected with indicated shRNA or plasmid, respectively. And then transwell assays were performed to determine the migration and the invasion of H1975 cells **(A)** and H460 cells **(C)**. Magnification, × 200. Three random fields of H1975 cells **(B)** and H460 cells **(D)** were photographed, and the cells in each field were calculated. Control, untreated cells; NC, scramble shRNA control. Data are presented as means ± *SD, n* = 3, ^***^p < 0.0001.

RETRACTED

Previous studies have demonstrated that cancer metastasis are partially dependent on the ability of tumor cells to adhere to the proteins of the extracellular matrix (ECM) and survive at the distant location (Glinsky and Glinsky, 1996; DeRoock et al., 2001), we thus examined the effects of HOXC10 on tumor cell adhesion to the ECM supportive substrate fibronectin using pre-coated plates (Mahauad-Fernandez et al., 2014). Compared with scrambled shRNA control, HOXC10 shRNA significantly reduced adhesive capability of H1975 cells to fibronectin (Figures 4A,C; *p* < 0.0001). In H460 cells, HOXC10 ectopic expression markedly enhanced the ability of cancer cells to adhere to fibronectin (Figures 4B,D; *p* < 0.0001). These results indicate that HOXC10 regulates adhesion of lung cancer cells to ECM proteins.

**Figure 4:** HOXC10 inhibits cell adhesion *in vitro*. H1975 cells and H460 cells were transfected with indicated shRNA or plasmid, respectively. Tumor cell adhesion assay was performed as described in materials and methods. Three random fields of H1975 cells **(A,C)** and H460 cells **(B,D)** were photographed, and the cells in each field were calculated. Magnification, × 200. Control, untreated cells; NC, scramble shRNA control. Data are presented as means ± *SD, n* = 3, ^***^p < 0.0001 vs. control group.

### HOXC10 regulates metastasis-related proteins expression

To further confirm HOXC10 was involved in regulating lung cancer metastasis on an unbiased basis, we performed gene set enrichment analysis (GSEA) using data from the TCGA dataset to detect coordinated differences in expression of predefined sets of functionally related genes. Metastasis-associated genes were identified with the significant association with high HOXC10 expression (Figure S1A). Thus, we further evaluated the phosphorylation level of PI3K, JNK, and ERK1/2 expression in response to HOXC10 interfere or overexpression. Western blotting analysis revealed that HOXC10 significantly increased phosphorylation level of PI3K, but not JNK or ERK1/2 (Figures 5A,B). As important downstream molecules of PI3K/AKT pathway and epithelial–mesenchymal transition (EMT) markers, matrix metalloproteinase (MMP) 2 and 9, Vascular cell adhesion molecule 1 (VCAM-1), vimentin and E-cadherin are involved in cancer metastasis (Hiratsuka et al., 2002; Larue and Bellacosa, 2005; Chen and Massague, 2012; Tang et al., 2014). The mRNA and protein levels of MMP-2, MMP-9, VCAM-1, and vimentin were decreased remarkably after being treated with HOXC10 shRNA compared to scrambled shRNA control or untreated H1975 cells, and E-cadherin was significantly enhanced in H1975 cells (Figures 5C,E, Figure S1B). As expected, HOXC10 ectopic expression in H460 cells markedly increased both mRNA and protein expressions of MMP-2, MMP-9, and VCAM-1, and inhibited E-cadherin expression (Figures 5D,F, Figure S1C). Overall, these findings suggest that high HOXC10 expression in human lung cancer tissues is correlated with metastasis.

RETRACTED

**Figure 5:** HOXC10 regulates expression of metastasis-related proteins in lung cancer cells. H1975 cells and H460 cells were transfected with indicated shRNA or plasmid, respectively. Forty eight hour later, western blotting analysis was performed to detect p-PI3K, PI3K, p-JNK, JNK, p-ERK1/2, ERK1/2, MMP-2/9, VCAM-1, vimentin, and E-cadherin expression in H1975 cells **(A,C)** and H460 cells **(B,D)**. mRNA expression of MMP-2/9, VCAM-1, vimentin and E-cadherin in H1975 cells **(E)** and H460 cells **(F)** was evaluated by qRT-PCR. GAPDH was used as internal control. Control, untreated cells; NC, scramble shRNA control. Data are presented as means ± *SD, n* = 3, ^**^p < 0.01; ^***^p < 0.0001.

### Upregulated HOXC10 expression indicates poor prognosis of lung cancer

Next, to support our conclusion that HOXC10 is upregulated in lung cancer, we further examined the expression of HOXC10 mRNA in lung cancer patients included in six GEO datasets (GSE19188, GSE31210, GSE10072, GSE7670, GSE32863, GSE30219). HOXC10 mRNA expression is significantly upregulated in cancer tissues of patients with lung adenocarcinoma, squamous cell carcinoma and small cell lung cancer than in normal lung tissues (Figures 6A,B). With the purpose to assess prognostic value of HOXC10, the patient samples in GSE30219 (with information of relapse free survival) were divided into two cohorts according to the median mRNA expression of HOXC10 (high vs. low expression). Patients with lung adenocarcinoma in the high HOXC10 expression subgroup showed worse relapse free survival compared to the low expression subgroup in GSE30219 (Figure 6C, *p* = 0.0062). However, the prognostic value of HOXC10 in lung squamous cell carcinoma (Figure 6D, *p* = 0.4125) and small cell lung cancer (Figure 6E, *p* = 0.0730) were not obvious as in lung adenocarcinoma, which may be limited by the small sample size of included patients. The prognostic significance of the mRNA expression of HOXC10 in lung adenocarcinoma and squamous cell carcinoma was further evaluated using the Kaplan-Meier plotter (www.kmplot.com), an online database including gene expression data and clinical data (Gyorffy et al., 2013). Similar with the results obtained from GSE30219, HOXC10 predicted a poor overall survival (Figure 6F, HR = 1.4, 95%CI:1.11–1.77, *p* = 0.0043) and relapse free survival (Figure 6G, HR = 1.4, 95%CI:1.02–1.96, *p* = 0.0366) of lung adenocarcinoma, but not obvious in lung squamous cell carcinoma (Figures 6H,I). Taken together, our data suggest that upregulated HOXC10 expression indicates poor survival and can be used as prognostic marker for the patients with lung cancer, especially for lung adenocarcinoma.

RETRACTED

**Figure 6:** Upregulated HOXC10 indicates poor survival of lung cancer patients. **(A)** The expression difference of HOXC10 between normal and lung cancer tissues in five GEO datasets (GSE19188, GSE31210, GSE10072, GSE7670, GSE32863, GSE30219), connection line means paired samples. **(B)** The expression of HOXC10 in lung cancer patients from GSE30219. **(C–E)** The Kaplan–Meier plot presents the relapse free survival of patients with lung adenocarcinoma (LUAD) **(C)**, Lung squamous cell carcinoma (LUSC) **(D)**, small cell lung cancer (SCLC) **(E)** in GSE30219. **(F–I)** Overall survival **(F)** and relapse free survival **(G)** curves were plotted for LUAD patients, Overall survival **(H)** and relapse free survival **(I)** curves were plotted for LUSC patients via the Kaplan–Meier plotter database. Patients with expression above the median are indicated in red line, and patients with expressions below the median in black line. HR means hazard ratio. Data are presented as means ± *SD*, ^**^p < 0.01; ^***^p < 0.0001.

## Discussion

Products of HOX genes are transcription factors responsible for regulating phenotype cell identity, differentiation, and controlling primary cellular processes (Care et al., 2001). Besides their function in embryonic development and tissue remodeling, HOX gene network has been well-described to involve in hematopoiesis and leukemogenesis (Argiropoulos and Humphries, 2007). Recently, inappropriate HOX gene expression has been associated with different neoplasias occurred in kidney, colon, lung, skin, bladder, liver, breast, and prostate (Cillo et al., 1992; Calvo et al., 2000; Abba et al., 2007; Cantile et al., 2009; Yuan et al., 2016). Specifically in lung cancer, several members of HOX gene family, like HOXA2, HOXB9, HOXA9, and HOXA10 were frequently up-regulated in lung cancer cell lines and direct tumors *in vivo* (Calvo et al., 2000; Plowright et al., 2009). In this study, we show for the first time, to our knowledge, that HOXC10 is crucial for cancer metastasis and its upregulation indicates a poor survival of lung adenocarcinoma patients from Wuhu No.2 People's Hospital, GEO datasets and Kaplan–Meier plotter database. Combined with the similar results that elevated HOXC10 expression is associated with increased invasiveness and indicates poor survival outcome of human cervical cancer and thyroid cancer (Zhai et al., 2007; Feng et al., 2015), our study further highlights the potential value of HOXC10 as a novel biomarker for human cancer prognosis evaluation.

RETRACTED

By comparing HOXC10 expression in clinical samples, we found that HOXC10 mRNA expression is significantly increased in human lung cancer tissues, especially in tissues from lung cancer patients with lymph node or distal metastasis. HOXC10 is upregulated following chemotherapy or ionizing radiation in ER-negative breast cancer. Then, as part of the Cdk-activating kinase complex, HOXC10 participates in the late stages of DNA repair that involves restart of transcription for recovery and survival of cancer cells in response to chemotherapy (Sadik et al., 2016). In this study, we noticed that patients with smoking history showed a higher level of HOXC10 expression than non-smokers, which may be attributed to tobacco smoking is one of the main causes of DNA damage (Cao et al., 2016) and the detailed molecular mechanisms of HOXC10 induction need to be investigated in future study.

In our study, HOXC10 expressed differently in five human lung cancer cell lines, H1975, PC-9, A549, H460, and H446. For example, H1975 cells has the highest level of HOXC10 expression, and H460 cells has the lowest. This inconsistency may be resulted by the intrinsic characteristics difference of different subtypes of human lung cancer, and traditional cell lines maintained in culture conditions are depart markedly from the natural setting of human cancers (Williams et al., 2013). To better unveil the roles of HOXC10 in lung cancer, patient-derived xenografts (PDX) models need to be used in future study. HOXC10 increased invasiveness of human cervical cancer–derived cell lines (Lopez et al., 2006) and expressed a relative higher level in metastatic breast cancer cell lines including MCF-7, MM361 and T47D (Pathiraja et al., 2014). Combined with the evidence that: (1) H1975 cells show higher lung tumorigenesis and metastasis potential than H460 cells (Wagner et al., 2013), (2) HOXC10 expression was significantly increased in lung adenocarcinoma patients with lymph node or distal metastasis, and predicted a poor survival of lung adenocarcinoma patients from our local hospital, GEO datasets and Kaplan–Meier plotter database, (3) Transient knockdown of HOXC10 expression inhibited migration and invasion of human thyroid cancer and reduced invasiveness of cervical carcinoma cells (Zhai et al., 2007; Feng et al., 2015), (4) our in-depth cellular study clearly demonstrate that HOXC10 promote metastasis of lung cancer cells *in vitro*. Thus, we could conclude that HOXC10 plays an important role in regulating lung cancer metastasis, at least in lung adenocarcinoma.

RETRACTED

Overexpression of HOXC10 activates PI3K and NF-κB pathways in human breast cancer and supports the development of chemotherapy resistance (Sadik et al., 2016). In this study, molecular analysis revealed that HOXC10 enhanced PI3K phosphorylation in lung cancer cells, and regulated EMT-related markers: MMP2, MMP9, VCAM-1, vimentin and E-cadherin expression in lung cancer cells both at mRNA and protein levels. Furthermore, we noticed that HOXC10 activated JNK and PI3K phosphorylation in lung adenocarcinoma cells, but not ERK1/2, which was activated in large cell lung cancer cells. Combined the different expression levels of HOXC10 in different lung cancer cell lines, the exact role of HOXC10 in different subtypes of lung cancer still needs a thorough investigation in future.

In conclusion, our study revealed that abnormal elevated expression of HOXC10 enhances migration, invasion and adhesion of lung cancer cells. With the observed clinical data that HOXC10 overexpresses in lung cancer tissues, especially in tissues with metastatic potential, and predicts a poor prognosis of lung cancer patients from our local hospital, GEO dataset, and Kaplan-Meier plotter database, our study may thus provide useful information for the development of HOX gene-targeted therapy or prognostic biomarker development.

## Author contributions

CY, ZC and TW conceived and coordinated the study, drafted and revised the manuscript. XT collected tissue samples and performed related qRT-PCR analysis. BD and YH performed cell culture and related experiments. HC performed Immunohistochemistry analysis. CY mined clinical and expression profile of HOXC10 from six GEO Datasets and Kaplan–Meier plotter database. All authors read and approved the final manuscript.

### Conflict of interest statement

The authors declare that the research was conducted in the absence of any commercial or financial relationships that could be construed as a potential conflict of interest. The reviewer XL and handling Editor declared their shared affiliation, and the handling Editor states that the process nevertheless met the standards of a fair and objective review.

## References

[B1] AbbaM. C.SunH.HawkinsK. A.DrakeJ. A.HuY.NunezM. I.. (2007). Breast cancer molecular signatures as determined by SAGE: correlation with lymph node status. Mol. Cancer Res. 5, 881–890. 10.1158/1541-7786.MCR-07-005517855657PMC4186709

RETRACTED

[B2] AlexanderT.NolteC.KrumlaufR. (2009). Hox genes and segmentation of the hindbrain and axial skeleton. Annu. Rev. Cell Dev. Biol. 25, 431–456. 10.1146/annurev.cellbio.042308.11342319575673

[B3] AnsariK. I.HussainI.KasiriS.MandalS. S. (2012). HOXC10 is overexpressed in breast cancer and transcriptionally regulated by estrogen via involvement of histone methylases MLL3 and MLL4. J. Mol. Endocrinol. 48, 61–75. 10.1530/JME-11-007822143955

[B4] ArgiropoulosB.HumphriesR. K. (2007). Hox genes in hematopoiesis and leukemogenesis. Oncogene 26, 6766–6776. 10.1038/sj.onc.121076017934484

[B5] CalvoR.WestJ.FranklinW.EricksonP.BemisL.LiE.. (2000). Altered HOX and WNT7A expression in human lung cancer. Proc. Natl. Acad. Sci. U.S.A. 97, 12776–12781. 10.1073/pnas.97.23.1277611070089PMC18840

[B6] CantileM.FrancoR.TschanA.BaumhoerD.ZlobecI.SchiavoG.. (2009). HOX D13 expression across 79 tumor tissue types. Int. J. Cancer 125, 1532–1541. 10.1002/ijc.2443819488988

[B7] CaoC.LaiT.LiM.ZhouH.LvD.DengZ.. (2016). Smoking-promoted oxidative DNA damage response is highly correlated to lung carcinogenesis. Oncotarget 7, 18919–18926. 10.18632/oncotarget.781026942876PMC4951340

[B8] CareA.FelicettiF.MecciaE.BotteroL.ParenzaM.StoppacciaroA.. (2001). HOXB7: a key factor for tumor-associated angiogenic switch. Cancer Res. 61, 6532–6539. 11522651

[B9] ChenK. N.GuZ. D.KeY.LiJ. Y.ShiX. T.XuG. W. (2005). Expression of 11 HOX genes is deregulated in esophageal squamous cell carcinoma. Clin. Cancer Res. 11, 1044–1049. 15709170

[B10] ChenM.HuW.XiongC. L.QuZ.YinC. Q.WangY. H.. (2016). miR-22 targets YWHAZ to inhibit metastasis of hepatocellular carcinoma and its down-regulation predicts a poor survival. Oncotarget 7, 80751–80764. 10.18632/oncotarget.1303727811373PMC5348352

[B11] ChenQ.MassagueJ. (2012). Molecular pathways: VCAM-1 as a potential therapeutic target in metastasis. Clin. Cancer Res. 18, 5520–5525. 10.1158/1078-0432.CCR-11-290422879387PMC3473104

[B12] CilloC.BarbaP.FreschiG.BucciarelliG.MagliM. C.BoncinelliE. (1992). Hox gene-expression in normal and neoplastic human kidney. Int. J. Cancer 51, 892–897. 10.1002/ijc.29105106101379214

[B13] DeRoockI. B.PenningtonM. E.SrokaT. C.LamK. S.BowdenG. T.BairE. L.. (2001). Synthetic peptides inhibit adhesion of human tumor cells to extracellular matrix proteins. Cancer Res. 61, 3308–3313. 11309285

[B14] FengX.LiT.LiuZ.ShiY.PengY. (2015). HOXC10 up-regulation contributes to human thyroid cancer and indicates poor survival outcome. Mol. Biosyst. 11, 2946–2954. 10.1039/C5MB00253B26279264

RETRACTED

[B15] FordeP. M.EttingerD. S. (2013). Targeted therapy for non-small-cell lung cancer: past, present and future. Expert Rev. Anticancer Ther. 13, 745–758. 10.1586/era.13.4723773106PMC3991462

[B16] GabelliniD.ColalucaI. N.VodermaierH. C.BiamontiG.GiaccaM.FalaschiA.. (2003). Early mitotic degradation of the homeoprotein HOXC10 is potentially linked to cell cycle progression. EMBO J. 22, 3715–3724. 10.1093/emboj/cdg34012853486PMC165610

[B17] GlinskyG. V.GlinskyV. V. (1996). Apoptosis amd metastasis: a superior resistance of metastatic cancer cells to programmed cell death. Cancer Lett. 101, 43–51. 10.1016/0304-3835(96)04112-28625281

[B18] GrierD. G.ThompsonA.KwasniewskaA.McGonigleG. J.HallidayH. L.LappinT. R. (2005). The pathophysiology of HOX genes and their role in cancer. J. Pathol. 205, 154–171. 10.1002/path.171015643670

[B19] GyorffyB.SurowiakP.BudcziesJ.LanczkyA. (2013). Online survival analysis software to assess the prognostic value of biomarkers using transcriptomic data in non-small-cell lung cancer. PLoS ONE 8:e82241. 10.1371/journal.pone.008224124367507PMC3867325

[B20] HamadaJ.OmatsuT.OkadaF.FuruuchiK.OkuboY.TakahashiY.. (2001). Overexpression of homeobox gene HOXD3 induces coordinate expression of metastasis-related genes in human lung cancer cells. Int. J. Cancer 93, 516–525. 10.1002/ijc.135711477555

[B21] HiratsukaS.NakamuraK.IwaiS.MurakamiM.ItohT.KijimaH.. (2002). MMP9 induction by vascular endothelial growth factor receptor-1 is involved in lung-specific metastasis. Cancer Cell 2, 289–300. 10.1016/S1535-6108(02)00153-812398893

[B22] ImielinskiM.BergerA. H.HammermanP. S.HernandezB.PughT. J.HodisE.. (2012). Mapping the hallmarks of lung adenocarcinoma with massively parallel sequencing. Cell 150, 1107–1120. 10.1016/j.cell.2012.08.02922980975PMC3557932

[B23] LarueL.BellacosaA. (2005). Epithelial-mesenchymal transition in development and cancer: role of phosphatidylinositol 3[prime] kinase//AKT pathways. Oncogene 24, 7443–7454. 10.1038/sj.onc.120909116288291

[B24] LopezR.GarridoE.VazquezG.PinaP.PerezC.AlvaradoI.. (2006). A subgroup of HOX Abd-B gene is differentially expressed in cervical cancer. Int. J. Gynecol. Cancer 16, 1289–1296. 10.1111/j.1525-1438.2006.00603.x16803519

[B25] MaL.WangR.NanY.LiW.WangQ.JinF. (2015). Phloretin exhibits an anticancer effect and enhances the anticancer ability of cisplatin on non-small cell lung cancer cell lines by regulating expression of apoptotic pathways and matrix metalloproteinases. Int. J. Oncol. 48, 843–853. 10.3892/ijo.2015.330426692364

[B26] MaX. J.SalungaR.TuggleJ. T.GaudetJ.EnrightE.McQuaryP.. (2003). Gene expression profiles of human breast cancer progression. Proc. Natl. Acad. Sci. U.S.A. 100, 5974–5979. 10.1073/pnas.093126110012714683PMC156311

RETRACTED

[B27] Mahauad-FernandezW. D.DemaliK. A.OlivierA. K.OkeomaC. M. (2014). Bone marrow stromal antigen 2 expressed in cancer cells promotes mammary tumor growth and metastasis. Breast Cancer Res. 16:493. 10.1186/s13058-014-0493-8PMC430884525499888

[B28] MiaoJ.WangZ.ProvencherH.MuirB.DahiyaS.CarneyE.. (2007). HOXB13 promotes ovarian cancer progression. Proc. Natl. Acad. Sci. U.S.A. 104, 17093–17098. 10.1073/pnas.070793810417942676PMC2040435

[B29] MorganR.PlowrightL.HarringtonK. J.MichaelA.PandhaH. S. (2010). Targeting HOX and PBX transcription factors in ovarian cancer. BMC Cancer 10:89. 10.1186/1471-2407-10-89PMC284688520219106

[B30] PathirajaT. N.NayakS. R.XiY.JiangS.GareeJ. P.EdwardsD. P.. (2014). Epigenetic reprogramming of HOXC10 in endocrine-resistant breast cancer. Sci. Transl. Med. 6, 229ra241. 10.1126/scitranslmed.300832624670685PMC4277862

[B31] PlowrightL.HarringtonK. J.PandhaH. S.MorganR. (2009). HOX transcription factors are potential therapeutic targets in non-small-cell lung cancer (targeting HOX genes in lung cancer). Br. J. Cancer 100, 470–475. 10.1038/sj.bjc.660485719156136PMC2658540

[B32] SadikH.KorangathP.NguyenN. K.GyorffyB.KumarR.HedayatiM.. (2016). HOXC10 expression supports the development of chemotherapy resistance by fine tuning DNA repair in breast cancer cells. Cancer Res. 76, 4443–4456. 10.1158/0008-5472.CAN-16-077427302171PMC4970943

[B33] ShahN.SukumarS. (2010). The Hox genes and their roles in oncogenesis. Nat. Rev. Cancer 10, 361–371. 10.1038/nrc282620357775

[B34] SiegelR.NaishadhamD.JemalA. (2013). Cancer statistics. Cancer J. Clin. 63, 11–30. 10.3322/caac.2116623335087

[B35] TangW.ZhuY.GaoJ.FuJ.LiuC.LiuY.. (2014). MicroRNA-29a promotes colorectal cancer metastasis by regulating matrix metalloproteinase 2 and E-cadherin via KLF4. Br. J. Cancer 110, 450–458. 10.1038/bjc.2013.72424281002PMC3899762

[B36] TiberioC.BarbaP.MagliM. C.ArveloF.Le ChevalierT.PouponM. F.. (1994). HOX gene expression in human small-cell lung cancers xenografted into nude mice. Int. J. Cancer 58, 608–615. 10.1002/ijc.29105804267914516

[B37] WagnerK. W.AlamH.DharS. S.GiriU.LiN.WeiY.. (2013). KDM2A promotes lung tumorigenesis by epigenetically enhancing ERK1/2 signaling. J. Clin. Invest. 123, 5231–5246. 10.1172/JCI6864224200691PMC3859406

[B38] WilliamsS. A.AndersonW. C.SantaguidaM. T.DyllaS. J. (2013). Patient-derived xenografts, the cancer stem cell paradigm, and cancer pathobiology in the 21st century. Lab. Invest. 93, 970–982. 10.1038/labinvest.2013.9223917877

[B39] WuX.ChenH.ParkerB.RubinE.ZhuT.LeeJ. S.. (2006). HOXB7, a homeodomain protein, is overexpressed in breast cancer and confers epithelial-mesenchymal transition. Cancer Res. 66, 9527–9534. 10.1158/0008-5472.CAN-05-447017018609

RETRACTED

[B40] YangY.AhnY. H.ChenY.TanX.GuoL.GibbonsD. L.. (2014). ZEB1 sensitizes lung adenocarcinoma to metastasis suppression by PI3K antagonism. J. Clin. Invest. 124, 2696–2708. 10.1172/JCI7217124762440PMC4038569

[B41] YuanC.ZhuX.HanY.SongC.LiuC.LuS.. (2016). Elevated HOXA1 expression correlates with accelerated tumor cell proliferation and poor prognosis in gastric cancer partly via cyclin D1. J. Exp. Clin. Cancer Res. 35, 1–16. 10.1186/s13046-016-0294-226791264PMC4721151

[B42] ZhaiY.KuickR.NanB.OtaI.WeissS. J.TrimbleC. L.. (2007). Gene expression analysis of preinvasive and invasive cervical squamous cell carcinomas identifies HOXC10 as a key mediator of invasion. Cancer Res. 67, 10163–10172. 10.1158/0008-5472.CAN-07-205617974957

